# Identification of Cardiac Patients Based on the Medical Conditions Using Machine Learning Models

**DOI:** 10.1155/2022/5882144

**Published:** 2022-07-20

**Authors:** Krishna Kumar, Narendra Kumar, Aman Kumar, Mazin Abed Mohammed, Alaa S. Al-Waisy, Mustafa Musa Jaber, Neeraj Kumar Pandey, Rachna Shah, Gaurav Saini, Fatma Eid, Mohammed Nasser Al-Andoli

**Affiliations:** ^1^Department of Hydro and Renewable Energy, Indian Institute of Technology, Roorkee 247667, India; ^2^School of Computing, DIT University, Dehradun 248009, Uttarakhand, India; ^3^AcSIR-Academy of Scientific and Innovative Research, Ghaziabad 201002, India; ^4^Structural Engineering Department, CSIR-Central Building Research Institute, Roorkee 247667, India; ^5^College of Computer Science and Information Technology, University of Anbar, Anbar 31001, Iraq; ^6^Computer Technologies Engineering Department, Information Technology Collage, Imam Ja'afar Al-Sadiq University, Baghdad, Iraq; ^7^Department of Computer Science, Dijlah University College, Baghdad, Iraq; ^8^Department of Medical Instruments Engineering Techniques, Al-Farahidi University, Baghdad 10021, Iraq; ^9^Department of CSE, Indian Institute of Information Technology, Guwahati 781015, India; ^10^Indian Institute of Engineering Science and Technology (IIEST), Shibpur, West Bengal 711103, India; ^11^Technology Management, College of Business, Stony Brook University, Stony Brook, NY, USA; ^12^Computer Science & Information Systems Department, Faculty of Science, Sa'adah University, Sa'adah, Yemen

## Abstract

Chronic diseases are the most severe health concern today, and heart disease is one of them. Coronary artery disease (CAD) affects blood flow to the heart, and it is the most common type of heart disease which causes a heart attack. High blood pressure, high cholesterol, and smoking significantly increase the risk of heart disease. To estimate the risk of heart disease is a complex process because it depends on various input parameters. The linear and analytical models failed due to their assumptions and limited dataset. The existing studies have used medical data for classification purposes, which help to identify the exact condition of the patient, but no one has developed any correlation equation which can be directly used to identify the patients. In this paper, mathematical models have been developed using the medical database of patients suffering from heart disease. Curve fitting and artificial neural network (ANN) have been applied to model the condition of patients to find out whether the patient is suffering from heart disease or not. The developed curve fitting model can identify the cardiac patient with accuracy, having a coefficient of determination (*R*^2^-value) of 0.6337 and mean absolute error (MAE) of 0.293 at a root mean square error (RMSE) of 0.3688, and the ANN-based model can identify the cardiac patient with accuracy having a coefficient of determination (*R*^2^-value) of 0.8491 and MAE of 0.20 at RMSE of 0.267, it has been found that ANN provides superior mathematical modeling than curve fitting method in identifying the heart disease patients. Medical professionals can utilize this model to identify heart patients without any angiography or computed tomography angiography test.

## 1. Introduction

Predicting cardiac sickness accurately may save someone's life, while an incorrect diagnosis can be deadly. Heart disease is made more likely by a host of risk factors, including high cholesterol, obesity, elevated triglyceride levels, and hypertension. Heart failure occurs when the heart's muscles fail to pump blood as efficiently as they should [1]. Shortness of breath may result from blood clots in the lungs. The heart weakens or stiffens over time due to certain cardiac conditions, such as restricted arteries in the heart or high blood pressure. People with heart disease may live longer if they get the proper treatment. A low-fat, low-sodium diet, 30 minutes of moderate exercise five days a week (or more), limiting alcohol, and quitting smoking use may all help lower your risk of heart disease. You may also be prescribed medications by your doctor if lifestyle changes aren't enough to keep your cardiac disease under control. If you have a cardiac condition, the medication you get will be tailored to your specific needs. Your doctor may recommend certain therapies or surgery if medication fails to work for you. The kind of heart illness and the degree of cardiac damage will dictate the type of surgery. These classic risk factors, such as a family history of early coronary artery disease, dyslipidemia, and age, are well documented in the etiological route of ischemic heart disease in women [1].

The prevention, diagnosis, and rehabilitation of humans with ischemic heart disease continue to be a major concern. A complex interplay of variables, including unique risk factors and disease pathogenesis for ischemic heart disease in women with nonobstructive coronary artery disease and coronary microvasculature and endothelium disorder, contribute to this conundrum. Chronic disease prediction is essential in healthcare informatics [2]. It is important to detect the sickness as soon as possible [3]. Heart disease and diabetes risk may be estimated using machine learning algorithms that analyze the data for these diseases. Medical, industrial, and educational domains can benefit from extracting valuable information from vast datasets via data mining. Machine learning (ML) is one of the fastest-growing fields of artificial intelligence [1, 4].

Cardiovascular disease is one of the leading causes of death. The current study focuses on detecting, altering, and addressing risk variables on an individual basis. Despite the fact that the incidence of various cardiovascular risk factors is increasing at different rates around the world, the magnitude of the increase has prompted researchers to look into the causes of the risk factors. This study's main purpose is to develop a model for detecting cardiac patients without using angiography or computed tomography angiography.

Heart disease may be detected in a variety of persons using machine-learning techniques. Neural networks (NN), decision trees (DT), CN2 rule inducers, Stochastic Gradient Descent, and support vector machine (SVM) were utilized, and found that the DT and SVM algorithms produce the best results in the 20-fold and 10-fold cross-validation tests 87.69% of the time [5]. Na et al. [6] developed an algorithm based on heart rate variability (HRV) to distinguish panic disorder from other types of anxiety. Because panic disorder and other anxiety disorders have similar causes and symptoms, machine learning aims to create a classification model that distinguishes panic disorder from other anxiety illnesses [6]. By finding complex, nonlinear patterns of expression and linkages in data sets, it has been found that the ML techniques may extract underlying information and found that for families, Random forest models yielded AUC values of more than 0.80, and for species, more than 0.98% [7]. The need for advanced tools to detect the illness early may reduce fatality rates. AI and data mining have many different methods that could help predict CVD before it happens and find out how people act in many different ways from a lot of data. The results of these forecasts will help doctors to make decisions and get patients checked out early, which will help them live longer. Different models can be utilized in several classification approaches [8].

Various researchers have developed a layered biometric identification system resistant to PAs by fusing fingerprint and heart-signal data. Artifact attacks are avoided in the first layer using an excellent convolutional neural network (CNN). An electrocardiography (ECG) image is used in the second layer of a lightweight CNN to prevent corpse attacks. Next, fingerprint matches at a predetermined threshold are utilized to prevent attacks by conformists. A score-level fusion of the fingerprint and a cardiac signal is used in the last layer of biometric authentication to ensure security. Two freely available online databases of fingerprints and cardiac signals were used to evaluate the proposed system against different scenarios of authentication and assault. There were no false match rates (FMRs) found in the experiments, and the false nonmatch rates were satisfactory (FNMR) [9]. A unique data-driven strategy with a fuzzy rule-based classification system for cardiac disease detection outperforms other models in order to balance interpretability and accuracy [10].

The prevalence of heart failure has been rising in lockstep with the pace of population growth [11]. A python-based app has been made for healthcare because it is more reliable and helps with the tracking and setting up different types of health monitoring Apps. A random forest classification system is being developed to diagnose cardiac problems. This method has an 83% of average accuracy rate over training data [12]. Dynamic systems (MLDS) have been developed to increase their existing knowledge at each layer. For feature selection, the model employs the correlation attribute evaluator (CAE), extra trees classifier (ETC), information gain attribute evaluator (IGAE), gain ratio attribute evaluator (GRAE), and Lasso. The ensemble approach for categorization in the model was built using random forest (RF), gradient boosting (GB), and naive Bayes (NB) classifiers [13].

Several statistical approaches, including principal component analysis, were used to find the essential parameters for stroke prediction. They have found that the most critical criteria for diagnosing stroke in patients are age, average glucose level, heart disease, and hypertension. Furthermore, compared to all accessible input characteristics and various benchmarking methodologies, a feed-forward neural network with four properties has the greatest accuracy rate and the lowest miss rate [14]. Three alternative goals have been chosen for CHF (chronic heart failure) modeling: CHF identification as the primary diagnostic, prediction of blood pressure, and classification of CHF stages. Several machine-learning algorithms were applied to three sorts of features for each job: static, dynamic, and the entire feature set. The findings suggest that the models perform better when temporal and nontemporal information are included [15]. Heart disease may be detected earlier because of the newly developed and improved algorithms that have been built, innovated, and optimized. Based on a variety of classifier algorithms, including NB, the salp swarm optimized neural network (SSA-NN), Bayesian optimized SVM (BO-SVM), and K-nearest neighbors, the created system for predicting cardiovascular illness have been put into practice (KNN) [16]. Heart failure models were used to analyze the severity of heart failure and predict the occurrence of adverse events such as destabilizations, re-hospitalizations, and death [17]. Total heart rate (HR) and ear-worn, long-term blood pressure (BP) monitor to improve wearability. An SVM classifier to learn and recognize raw heartbeats from moving artifact-influenced data [18]. A single mechanocardiography measurement and the atrial fib relation (AFib) can be correctly identified acute decompensated heart failure can be diagnosed with a reasonable level of accuracy [19].

Machine learning establishes a new technique for detecting significant features which enhance the accuracy of the prediction of cardiovascular disease. A hybrid random forest and linear model approach improve the performance while maintaining an accuracy rate of 88.7% in predicting heart disease [20]. Enhanced deep learning assisted convolutional neural network algorithm was used to help and enhance patient prognostics in heart disease. It has been added to the IoMT for expert systems that help clinicians quickly and efficiently diagnose cardiac patients' information on cloud platforms worldwide. Compared to standard techniques, the test findings suggest that if you have a lot of flexibility with your EDCNN hyperparameters, you can get an accuracy of up to 99.1%. A unique rapid conditional mutual information feature selection approach has been developed to overcome the feature selection challenges [21].

The feature selection methods were used for feature selection in order to improve classification accuracy and minimize classification system execution time. The experimental findings suggest that the feature selection method (FCMIM) may be used with a classifier support vector machine to create a high-level intelligent system to detect heart disease [22]. Heart rate variability is a powerful predictor of hypertensive individuals who are more likely to experience cardiovascular-related events. In contrast to the standard methodologies utilized for the same purpose, the supervised learning model is simple, efficient, and cost-effective, and it can be used for cardiac monitoring analysis [23]. Various researchers have used machine-learning algorithms to predict the ECG signals [24, 25]. As we mentioned, ML techniques can be applied in different applications and used especially in medical identification [26–28].

The medical field has a massive amount of patient data. This data must be mined using different machine-learning methods. Healthcare experts analyze this data in order to make effective diagnostic decisions. Clinical help can be provided by analyzing medical data using classification algorithms. The existing studies have used medical data for classification purposes which help to identify the exact condition of the patient, but no one has developed any correlation equation which can be directly used to identify the patients. In this study, basic information with some important clinical data have been used to identify the cardiac patient at the early stage without going through angiography and CT angiography. The major contributions of this study are the following:

- The correlation has been developed using curve fitting and artificial neural network (ANN) methods.
- Developed an artificial neural network (ANN) model that professionals can use to identify cardiac patients. An ANN-based model provides results with very high accuracy.
- A detailed discussion on heart disease and a selective literature review has been done to identify the issues and parameters related to the cardiac disease for testing and identification purposes.
- The data has been collected from the Kaggle database. The performance of the models has been compared. The results show that these correlations can help in identify cardiac patients easily with higher precision.

The rest of the paper is organized in the following sections.  Section 2 presents the details of data collection and data preparation which has been used for modeling. The correlation models using curve fitting and artificial neural network methods are presented in Section 3. The major findings and performance of the models of curve fitting and ANN models are summarized in Section 4.

## 2. Cardiac Patients Identification

Identification of cardiac patients in the early stages is important to reduce the risk of complications. To address this issue, it is proposed to develop correlations that can be utilized to identify cardiac patients. A methodology has been proposed, as shown in Figure 1. The data sets have been collected from the online database, and the data filtration and standardization operations have been performed to remove outliers and make the data dimensionless. The proposed curve fitting and ANN methods have been used to develop models, and the performance of the developed models has been tested on various performance parameters to select the best-fitted model.

### 2.1. Data Collection and Data Preparation

The clinical parameters of a heart disease patient were collected from the open-source link (https://github.com/g-shreekant/Heart-Disease-Prediction-using-Machine-Learning) used for the development of correlation [29]. A list of such parameters is listed in Table 1. For the modeling of parameters, all the parameter values are standardized in the range of 0 to 1 using equation (1). The details of the statistical properties of the parameters used for the modeling are listed in Table 2 to understand the features of the data.  Figure 2 shows the correlation plot between the input (*X*) and output (*Y*) variables.

(1) $$\begin{array}{c} Y=\frac{\left(X-X_{\text{min}}\right)}{X_{\text{max}}-X_{\text{min}}}, \end{array}$$

where *Y* is the output of the normalized value, *x* is the value to be normalized, *X*_min_ is the minimum value in the selected dataset, and *X*_max_ is the maximum value in the selected dataset.

Shapley additive explanations (SHAP) of the input parameters considered for modeling are shown in Figure 3. It is used to determine the contribution of each input parameter in the final predicted output. It shows that the thalassemia value (*T*_*h*_) is the most important parameter and fasting blood sugar (*F*_*b*_) is the least important parameter in predicting a heart patient. The relevance of every variable can be determined based on the SHAP values. The red dot indicates that the feature value is high, which leads to a higher SHAP value.

The detailed methodology of the proposed work for the identification of cardiac patients based on the medical conditions using machine-learning models is given in Figure 3.

## 3. Modeling of Parameters

The predicted value of the heart disease patient equation can be written as follows:

(2) $$\begin{array}{c} H_{d}=f\left(A_{c},S_{c},C_{p},B_{p},C_{h},F_{b},R_{e},H_{r},E_{x},O_{p},S_{p},C_{a},T_{h}\right). \end{array}$$

### 3.1. Curve Fitting Technique

The relationship between the predicted heart disease value (*H*_*d*_) and patient age (*A*_*c*_) is shown in Figure 4, and equation (3) shows the relationship between *H*_*d*_ and *A*_*c*_:

(3) $$\begin{array}{c} H_{d}=-0.0123A_{c}+1.2152. \end{array}$$

Let *A*_0_=1.2152, and the values *A*_*0*_ depend on other input parameters such as *S*_*c*_, *C*_*p*_, *B*_*p*_, *C*_*h*_, *F*_*b*_, *R*_*e*_, *H*_*r*_, *E*_*x*_, *O*_*p*_, *S*_*p*_, *C*_*a,*_ and *T*_*h*_.

Equation (3) can be written as follows:

(4) $$\begin{array}{c} H_{d}=-0.0123A_{c}+A_{0}. \end{array}$$

We can rewrite the (4) as follows:

(5) $$\begin{array}{c} A_{0}=H_{d}+0.0123A_{c}. \end{array}$$

Figure 5 shows the plot between *A*_0_ and *S*_*c*_, and the relationship between *A*_0_ and *S*_*c*_ is expressed in equation (6):

(6) $$\begin{array}{c} A_{0}=-0.3069S_{c}+0.7647. \end{array}$$

Let *B*_0_=0.7647, the value of *B*_0_ depends on other input parameters such as *C*_*p*_, *B*_*p*_, *C*_*h*_, *F*_*b*_, *R*_*e*_, *H*_*r*_, *E*_*x*_, *O*_*p*_, *S*_*p*_, *C*_*a*_, and *T*_*h*_.

Equation (6) can be written as follows:

(7) $$\begin{array}{c} A_{0}=-0.3069S_{c}+B_{0}. \end{array}$$

We can rewrite the equation (7) as follows:

(8) $$\begin{array}{c} B_{0}=A_{0}+0.3069S_{c}. \end{array}$$

Figure 6 shows the plot between *B*_0_ and *C*_*p*_, and the relationship between *B*_0_ and *C*_*p*_ is expressed in equation (9):

(9) $$\begin{array}{c} B_{0}=0.606C_{p}+0.5688. \end{array}$$

Consider, *C*_0_=0.5688, and it also depends on other input parameters such as *B*_*p*_, *C*_*h*_, *F*_*b*_, *R*_*e*_, *H*_*r*_, *E*_*x*_, *O*_*p*_, *S*_*p*_, *C*_*a*_, and *T*_*h*_.

Equation (9) can be written as follows:

(10) $$\begin{array}{c} B_{0}=0.606C_{p}+C_{0}. \end{array}$$

We can re-write the (10) as follows:

(11) $$\begin{array}{c} C_{0}=B_{0}-0.606C_{p}. \end{array}$$

Figure 7 shows the plot between *C*_0_ and *B*_*p*_, and the relationship between *C*_0_ and *B*_*p*_ is expressed in equation (12):

(12) $$\begin{array}{c} C_{0}=-0.544B_{p}+0.7619. \end{array}$$

Consider, *D*_0_=0.7619, this value also depends on other input parameters such as *C*_*h*_, *F*_*b*_, *R*_*e*_, *H*_*r*_, *E*_*x*_, *O*_*p*_, *S*_*p*_, *C*_*a,*_ and *T*_*h*_.

Equation (12) can be written as follows:

(13) $$\begin{array}{c} C_{0}=-0.544B_{p}+D_{0}. \end{array}$$

We can rewrite the (13) as follows:

(14) $$\begin{array}{c} D_{0}=C_{0}+0.544B_{p}. \end{array}$$

Figure 8 shows the plot between *D*_0_ and *C*_*h*_, and the relationship between *D*_0_ and *C*_*h*_ is expressed in equation (15):

(15) $$\begin{array}{c} D_{0}=-0.3923C_{h}+0.87. \end{array}$$

Let *E*_0_=0.87, the constant value *D*_0_ also depends on other input parameters such as *F*_*b*_, *R*_*e*_, *H*_*r*_, *E*_*x*_, *O*_*p*_, *S*_*p*_, *C*_*a,*_ and *T*_*h*_.

Equation (15) can be written as follows:

(16) $$\begin{array}{c} D_{0}=-0.3923C_{h}+E_{0}. \end{array}$$

We can rewrite the (16) as follows:

(17) $$\begin{array}{c} E_{0}=D_{0}+0.3923C_{h}. \end{array}$$

Figure 9 shows the plot between *E*_0_ and *F*_*b*_, and the relationship between *E*_0_ and *F*_*b*_ is expressed in equation (18):

(18) $$\begin{array}{c} E_{0}=-0.0336F_{b}+0.875. \end{array}$$

Consider, *F*_0_=0.875, this constant value also depends on other input parameters such as *R*_*e*_, *H*_*r*_, *E*_*x*_, *O*_*p*_, *S*_*p*_, *C*_*a*_, and *T*_*h*_.

Equation (18) can be written as follows:

(19) $$\begin{array}{c} E_{0}=-0.0336F_{b}+F_{0}. \end{array}$$

We can rewrite the (19) as follows:

(20) $$\begin{array}{c} F_{0}=E_{0}+0.0336F_{b}. \end{array}$$

Figure 10 shows the plot between *F*_0_ and *R*_*e*_, and the relationship between *F*_0_ and *R*_*e*_ is expressed in equation (21):

(21) $$\begin{array}{c} F_{0}=0.1179R_{e}+0.8439. \end{array}$$

Consider, *G*_0_=0.8439, this constant value also depends on other input parameters such as *H*_*r*_, *E*_*x*_, *O*_*p*_, *S*_*p*_, *C*_*a,*_ and *T*_*h*_.

Equation (21) can be written as follows:

(22) $$\begin{array}{c} F_{0}=0.1179R_{e}+G_{0}. \end{array}$$

We can rewrite the equation (22) as follows:

(23) $$\begin{array}{c} G_{0}=F_{0}-0.1179R_{e}. \end{array}$$

Figure 11 shows the plot between *G*_0_ and *H*_*r*_, and the relationship between *G*_0_ and *H*_*r*_ is expressed in equation (24):

(24) $$\begin{array}{c} G_{0}=0.7868H_{r}+0.3717. \end{array}$$

Consider, *H*_0_=0.3717, this constant value also depends on other input parameters such as *E*_*x*_, *O*_*p*_, *S*_*p*_, *C*_*a*_, and *T*_*h*_.

Equation (24) can be written as follows:

(25) $$\begin{array}{c} G_{0}=0.7868H_{r}+H_{0}. \end{array}$$

We can rewrite the (25) as follows:

(26) $$\begin{array}{c} H_{0}=G_{0}-0.7868H_{r}. \end{array}$$

Figure 12 shows the plot between *H*_0_ and *E*_*x*_, and the relationship between *H*_0_ and *E*_*x*_ is expressed in equation (27):

(27) $$\begin{array}{c} H_{0}=-0.1128E_{x}+0.408. \end{array}$$

Consider, *I*_0_=0.408, this constant value also depends on other input parameters such as *O*_*p*_, *S*_*p*_, *C*_*a*_, and *T*_*h*_.

Equation (27) can be written as follows:

(28) $$\begin{array}{c} H_{0}=-0.1128E_{x}+I_{0}. \end{array}$$

We can rewrite the (28) as follows:

(29) $$\begin{array}{c} I_{0}=H_{0}+0.1128E_{x}. \end{array}$$

Figure 13 shows the plot between *I*_0_ and *O*_*p*_, and the relationship between *I*_0_ and *O*_*p*_ is expressed in equation (30):

(30) $$\begin{array}{c} I_{0}=-0.4702O_{p}+0.4871. \end{array}$$

Consider, *J*_0_=0.4871, this constant value also depends on other input parameters such as *S*_*p*_, *C*_*a*_, and *T*_*h*_.

Equation (30) can be written as follows:

(31) $$\begin{array}{c} I_{0}=-0.4702O_{p}+J_{0}. \end{array}$$

We can rewrite the (31) as follows:

(32) $$\begin{array}{c} J_{0}=I_{0}+0.4702O_{p}. \end{array}$$

Figure 14 shows the plot between *J*_0_ and *S*_*p*_, and the relationship between *J*_0_ and *S*_*p*_ is expressed in equation (33):

(33) $$\begin{array}{c} J_{0}=0.0258S_{p}+0.469. \end{array}$$

Let *K*_0_=0.469, the constant value *K*_*0*_ also depends on other input parameters such as *C*_*a*_ and *T*_*h*_.

Equation (33) can be written as follows:

(34) $$\begin{array}{c} J_{0}=0.0258S_{p}+K_{0}. \end{array}$$

We can re-write the (34) as follows:

(35) $$\begin{array}{c} K_{0}=J_{0}-0.0258S_{p}. \end{array}$$

Figure 15 shows the plot between *K*_0_ and *C*_*a*_, and the relationship between *K*_0_ and *C*_*a*_ is expressed in equation (36):

(36) $$\begin{array}{c} K_{0}=-0.2628C_{a}+0.5168. \end{array}$$

Let *L*_0_=0.5168, and the constant value *L*_0_ only depends on one input parameter, that is *T*_*h*_.

Equation (36) can be written as follows:

(37) $$\begin{array}{c} K_{0}=-0.2628C_{a}+L_{0}. \end{array}$$

We can rewrite the (37) as follows:

(38) $$\begin{array}{c} L_{0}=K_{0}+0.2628C_{a}. \end{array}$$

Figure 16 shows the plot between *L*_0_ and *T*_*h*_, and the relationship between *L*_0_ and *T*_*h*_ is expressed in equation (39):

(39) $$\begin{array}{c} L_{0}=-0.2223T_{h}+0.6861. \end{array}$$

Let, *M*_0_=0.6861

Equation (39) can be written as follows:

(40) $$\begin{array}{c} L_{0}=-0.2223T_{h}+M_{0}. \end{array}$$

We can rewrite the (40) as follows:

(41) $$\begin{array}{c} M_{0}=L_{0}+0.2223T_{h}. \end{array}$$

Solving equations (5), (8), (11), (14), (17), (20), (23), (26), (29), (32), (35), (38), and (41) to find out *H*_*d*_.

(42) $$\begin{array}{c} H_{d}=M_{0}-0.0123A_{c}-0.3069S_{c}+0.606C_{p}-0.544B_{p}\\ -0.3923C_{h}-0.0336F_{b}+0.1179R_{e}+0.7868H_{r}\\ -0.1128E_{x}-0.4702O_{p}+0.0258S_{p}-0.2628C_{a}-0.2223T_{h}. \end{array}$$

Equation (42) can be utilized for identifying the heart disease patient.  Figure 17 shows a comparison between the predicted behavior and reported through the medical test. At an average value of *M*_0_, that is, 0.6881. The curve fitting method can predict heart disease patients with *R*^2^-the value of 0.6337, with a mean absolute error of 0.293 at RMSE of 0.3688. The curve fitting method gives poor performance; hence, it cannot use for prediction purposes.

### 3.2. ANN Technique

In 1944, Walter Pitts and Warren McCullough developed new types of networks called neural networks. One of the most extensively used machines learning approaches is the artificial neural network (ANN) model, which is inspired by biological neurons. The ANN is the most commonly used statistical model for detecting the relationship between input and output via a set of interconnected data structures with multiple neurons capable of enormous calculations for information representation and data processing. ANN model might be trained to forecast the required output from the supplied input. ANN is a type of artificial intelligence that operates in the same way as the human brain. ANN is made up of a sequence of linked neurons stacked in layers, just like the human brain. The weights linking the neurons determine the capacity of ANN structures to process provided information. The ANN structure can be either feed-forward or recurrent; however, feedforward is the most commonly employed in engineering and also utilized in this study. The feedforward network is made up of three layers: input, hidden, and output layer, as shown in Figure 18. The neurons in the same layer cannot be connected with each other, but they are also connected to the adjacent layers. Neurons are linked together and have different weights. Gradient descent and backpropagation are generally implemented to decrease errors. This method separated the data into three sections on a random basis: 90% for training, 5% for validation, and 5% for testing; the same approach is employed in this investigation. TANSIG (43) and PURELIN (34) were chosen as the activation functions in the hidden and output layers, respectively.

(43) $$\begin{array}{c} y=\text{tansig}\left(x\right)\\ =\frac{2}{\left(1+e^{-2x}\right)}-1, \end{array}$$

(44) $$\begin{array}{c} y=\text{purlin}\left(x\right)\\ =x. \end{array}$$

ANN is one of the popular machine-learning techniques utilized to predict heart disease patients. A total of 303 samples were employed to model the parameters, with 90% of the data architecture used for training, 5% used for validation, and 5% used for testing. Only a single hidden layer with neurons from 5 to 25 was used to obtain the best network. The hit-and-trial approach was applied to the performance indices (R and MSE) to calculate the ranking of training, testing, and validation datasets. The training, testing, and validation datasets' ranking results reveal that the 10 neurons in the hidden layer have the best performance.

The error ratio plot presented in (Figure 19(a)) and the performance plot (Figure 19(b)) using the ANN model at a minimum MSE of 0.08781 has been obtained at the 12 iterations.  Figure 19(c) depicts the learning process for the best-analyzed neural network gradient, momentum, and validation check. The detailed histogram of the training, validation, and testing of input data is shown in Figure 20.

The following is the mathematical expression between the standardized input parameters and the output:

(45) $$\begin{array}{c} H_{d}=f_{n}\left\{b_{0}+\sum_{k=1}^{h}\left[w_{k}f_{n}\left(b_{hk}+\sum_{i=1}^{m}w_{ik}X_{i}\right)\right]\right\}. \end{array}$$

The heart disease patient can be predicted using the equation (43). If the value of *H*_*d*_ is equal to 1 shows the patient has heart disease, and if the value is 0, then the patient is not suffering from heart disease:

(46) $$\begin{array}{c} H_{d}=1.35A_{1}+1.22A_{2}-1.26A_{3}+1.44A_{4}+-1.39A_{5}-0.87A_{6}+0.39A_{7}+0.58A_{8}-0.74A_{9}-0.77A_{10}+3\text{.}38\text{,} \end{array}$$

where the hidden neuron responses *A*_*i*_ (*i* = 1 to 10) are fed to the network output value and can be calculated with the equation (47).

(47) $$\begin{array}{c} \left[\begin{array}{c} A_{1}\\ A_{2}\\ A_{3}\\ A_{4}\\ A_{5}\\ A_{6}\\ A_{7}\\ A_{8}\\ A_{9}\\ A_{10} \end{array}\right]=\text{Tansig}\left(\left(\left[\begin{array}{ccccccccccccc} 0.26 & 0.20 & -0.49 & 0.32 & 0.16 & -0.58 & 0.89 & 0.36 & -0.81 & -0.76 & -1.12 & 1.29 & 0.07\\ -3.39 & 0.95 & 0.19 & -3.80 & -2.15 & -0.68 & -0.64 & 0.19 & -0.07 & -0.80 & 0.24 & 1.09 & 0.95\\ -3.20 & 1.35 & 0.73 & -3.27 & -0.79 & -0.13 & -0.52 & 0.31 & -0.47 & -0.23 & 0.32 & 1.95 & 0.03\\ 0.63 & 1.58 & 0.39 & -0.56 & 1.80 & 0.31 & 0.06 & -0.96 & -0.49 & 0.34 & 0.62 & 0.98 & 1.12\\ 1.55 & 1.57 & 0.27 & -1.79 & -0.00 & -1.01 & -0.69 & -1.21 & 2.26 & 0.13 & -1.09 & 0.89 & 0.09\\ -2.46 & -1.44 & 0.08 & 0.85 & 0.48 & -0.97 & 0.29 & -0.28 & -2.93 & -0.87 & 1.15 & 2.29 & 0.29\\ -1.34 & -1.86 & 2.47 & -0.11 & -1.51 & -0.19 & -0.29 & -0.95 & 0.76 & -0.86 & -0.32 & -1.09 & -0.00\\ 0.15 & 1.79 & 0.39 & -1.13 & 1.60 & -1.37 & -0.82 & -2.22 & 0.81 & 0.48 & 0.22 & 1.27 & -0.92\\ 1.07 & 0.01 & 1.23 & -2.26 & -0.49 & 0.85 & -1.34 & 1.79 & -0.38 & -0.89 & 2.67 & -2.19 & -4.38\\ 0.93 & -0.19 & -1.14 & -1.31 & 1.33 & -0.37 & 0.69 & 0.43 & 0.25 & -0.31 & 2.25 & 0.33 & -0.39 \end{array}\right]\times \left[\begin{array}{c} A_{c}\\ S_{c}\\ C_{p}\\ B_{p}\\ C_{h}\\ F_{b}\\ R_{e}\\ H_{r}\\ E_{x}\\ O_{p}\\ S_{p}\\ C_{a}\\ T_{h} \end{array}\right]\right)+\left[\begin{array}{c} -1.62\\ -2.91\\ 0.01\\ -2.93\\ 1.32\\ -1.34\\ -0.89\\ 2.39\\ -1.14\\ 3.49 \end{array}\right]\right). \end{array}$$

As shown in Figure 20, the final correlation can predict the patient with an *R*^2^-value of 0.8491, having an average mean absolute error of 0.20 at 0.267 of RMSE. As a result, it has been determined that the generated correlation indicated by (44) is the best for predicting the heart disease patient. As shown in Figure 21, the maximum values of the output parameter only lie on the two points that are 0 and 1. The proposed model is good for forecasting the diseases of heart patients.

## 4. Conclusion

Heart disease is one of the dangerous chronic diseases in which patient lives at the risk of heart attack or sometimes death. The current study generated an efficient correlation for identifying heart disease patients. Curve fitting and ANN were applied to the normalized medical results to develop the correlations. The key finding of this investigation is the curve fitting method-based correlation is not suitable for identifying the heart disease patient as its accuracy is low. The curve fitting method predicts with *R*^2^-value 0.6337 having a mean absolute error of 0.293 at RMSE of 0.3688. The ANN-based correlation can identify the heart disease patient with the coefficient of determination of 0.8491, having an average MAE of 0.20 at 0.267 of RMSE. The ANN-based developed correlation method is accurate for identifying the heart disease patient. This model can be utilized to identify the heart disease patient without the need for angiography or computed tomography angiography test.

## Figures and Tables

**Figure 1:** Methodology of the proposed work.

**Figure 2:** Correlation plot between input and output parameter.

**Figure 3:** Feature importance: (a) SHAP feature importance measured as the mean absolute shapley values; (b) variable importance plot; (c) SHAP summary plot.

**Figure 4:** Relationship plot of *H*_*d*_ vs. *A*_*c*_.

**Figure 5:** Relationship plot of *A*_*o*_ vs. *B*_*p*_.

**Figure 6:** Relationship plot of *B*_*o*_ vs. *C*_*p*_.

**Figure 7:** Relationship plot of *C*_*o*_ vs. *B*_*p*_.

**Figure 8:** Relationship plot of *D*_*o*_ vs. *C*_*h*_.

**Figure 9:** Relationship plot of *E*_*o*_ vs. *F*_*b*_.

**Figure 10:** Relationship plot of *F*_*o*_ vs. *R*_*e*_.

**Figure 11:** Relationship plot of *G*_*o*_ vs. *H*_*r*_.

**Figure 12:** Relationship plot of *H*_*o*_ vs. *E*_*x*_.

**Figure 13:** Relationship plot of *Io* vs. *O*_*p*_.

**Figure 14:** Relationship plot of *J*_*o*_ vs. *S*_*p*_.

**Figure 15:** Relationship plot of *K*_*o*_ vs. *C*_*a*_.

**Figure 16:** Relationship plot of *L*_*o*_ vs. *T*_*h*_.

**Figure 17:** A comparison between the predicted behavior and reported through the medical test.

**Figure 18:** Structure of ANN.

**Figure 19:** (a) Histogram of training, testing, and validation data. (b) Performance plot. (c) Learning process.

**Figure 20:** Results of ANN model: (a) Training data, (b) validation data, (c) testing data, and (d) all data.

**Figure 21:** Results obtained from ANN.

**Table 1:** Statistical data for every major parameter in the study.

S. No.	Parameter	Symbol	Description
1.	Age	*A*_*c*_	Years
2.	Sex	*S*_*c*_	1 = male, 0 = female
3.	Chest pain type	*C*_*p*_	Value 1: atypical angina, value 2: non-anginal pain, value 3: typical angina
4.	Blood pressure	*B*_*p*_	mm Hg on admission to the hospital
5.	Cholesterol	*C*_*h*_	mg/dl
6.	Fasting blood sugar	*F*_*b*_	>120 mg/dl, 1 = true; 0 = false
7.	Resting electrocardiographic results	*R*_*e*_	Value 0: probable, value 1: normal, value 2: having ST-T wave abnormality
8.	Maximum heart rate	*H*_*r*_	BPM
9.	Exercise-induced angina	*E*_*x*_	1 = yes; 0 = no
10.	ST depression induced by exercise relative to rest	*O*_*p*_	—
11.	The slope of the peak exercise ST segment	*S*_*p*_	0: downsloping; 1: flat; 2: upsloping 0: down sloping; 1: flat; 2: upsloping
12.	The number of significant vessels	*C*_*a*_	(0–3)
13.	Thalassemia value	*T*_*h*_	Value 1: fixed defect, value 2: normal blood flow, value 3: reversible defect

**Table 2:** Statistical properties of the medical data.

	Parameters												
	*A*_*c*_	*S*_*c*_	*C*_*p*_	*B*_*p*_	*C*_*h*_	*F*_*b*_	*R*_*e*_	*H*_*r*_	*E*_*x*_	*O*_*p*_	*S*_*p*_	*C*_*a*_	*T*_*h*_
Maximum	1.00	1.00	1.00	1.00	1.00	1.00	1.00	1.00	1.00	1.00	1.00	1.00	1.01
Minimum	0.00	0.00	0.00	0.00	0.00	0.00	0.00	0.00	0.00	0.00	0.00	0.00	0.00
Mean	0.32	0.36	0.28	0.15	0.26	0.60	0.33	0.17	0.70	0.18	0.77	0.55	0.55
Median	0.33	0.34	0.26	0.00	0.50	0.63	0.00	0.13	0.50	0.00	0.67	1.00	1.00
Mode	0.00	0.25	0.18	0.00	0.50	0.69	0.00	0.00	1.00	0.00	0.67	1.00	0.01
Range	1.00	1.00	1.00	1.00	1.00	1.00	1.00	1.00	1.00	1.00	1.00	1.00	1.01
Std.	0.34	0.17	0.12	0.36	0.26	0.17	0.47	0.19	0.31	0.26	0.20	0.50	0.50
Skewness	0.48	0.71	1.18	1.98	0.16	−0.54	0.75	1.27	−0.52	1.31	−0.48	−0.19	−0.19
Kurtosis	−1.20	0.90	4.59	1.92	−1.36	−0.03	−1.45	1.56	−0.62	0.83	0.30	−1.98	−1.98

## Data Availability

The clinical parameters of a heart disease patient were collected from the open-source link (https://github.com/g-shreekant/Heart-Disease-Prediction-using-Machine-Learning) used for the development of correlation.

## Notation

*A*_*c*_: Age
*S*_*c*_: Sex
*C*_*p*_: Chest pain type
*B*_*p*_: Blood pressure
*C*_*h*_: Cholesterol
*F*_*b*_: Fasting blood sugar
*R*_*e*_: Resting electrocardiographic results
*H*_*r*_: Maximum heart rate
*E*_*x*_: Exercise-induced angina
*O*_*p*_: ST depression induced by exercise relative to rest
*S*_*p*_: The slope of the peak exercise ST segment
*C*_*a*_: The number of significant vessels
*T*_*h*_: Thalassemia value
R: Correlation coefficient
*R* ^2^: Coefficient of determination
MSE: Mean square error
SSA-NN: Salp swarm optimized neural network
BO-SVM: Bayesian optimized SVM
AFib: Atrial fib relation
SHAP: Shapley additive explanations

### Anonyms

CAD: Coronary artery disease
ANN: Artificial neural network
RMSE: Root mean square error
ML: Machine learning
NN: Neural networks
DT: Decision trees
SVM: Support vector machine
HRV: Heart rate variability
CNN: Convolutional neural network
CAE: correlation attribute evaluator
ETC: Extra trees classifier
IGAE: Information gain attribute evaluator
GRAE: Gain ratio attribute evaluator
RF: Random forest
GB: Gradient boosting
NB: Naive Bayes
HF: Chronic Heart Failure
BP: Blood pressure
MAE: Mean absolute error.
